RETRACTED

# MMP-9, uPAR and Cathepsin B Silencing Downregulate Integrins in Human Glioma Xenograft Cells *In Vitro* and *In Vivo* in Nude Mice

**DOI:** 10.1371/journal.pone.0011583

**Published:** 2010-07-15

**Authors:** Krishna Kumar Veeravalli, Chandramu Chetty, Shivani Ponnala, Christopher S. Gondi, Sajani S. Lakka, Daniel Fassett, Jeffrey D. Klopfenstein, Dzung H. Dinh, Meena Gujrati, Jasti S. Rao

**Affiliations:** 1 Department of Cancer Biology and Pharmacology, University of Illinois College of Medicine at Peoria, Peoria, Illinois, United States of America; 2 Department Neurosurgery, University of Illinois College of Medicine at Peoria, Peoria, Illinois, United States of America; 3 Department Pathology, University of Illinois College of Medicine at Peoria, Peoria, Illinois, United States of America; Dresden University of Technology, Germany

## Abstract

**Background:**

Involvement of MMP-9, uPAR and cathepsin B in adhesion, migration, invasion, proliferation, metastasis and tumor growth has been well established. In the present study, MMP-9, uPAR and cathepsin B genes were downregulated in glioma xenograft cells using shRNA plasmid constructs and we evaluated the involvement of integrins and changes in their adhesion, migration and invasive potential.

**Methodology/Principal Findings:**

MMP-9, uPAR and cathepsin B single shRNA plasmid constructs were used to downregulate these molecules in xenograft cells. We also used MMP-9/uPAR and MMP-9/cathepsin B bicistronic constructs to evaluate the cumulative effects. MMP-9, uPAR and cathepsin B downregulation significantly inhibits xenograft cell adhesion to several extracellular matrix proteins. Treatment with MMP-9, uPAR and cathepsin B shRNA of xenografts led to the downregulation of several alpha and beta integrins. In all the assays, we noticed more prominent effects with the bicistronic plasmid constructs when compared to the single plasmid shRNA constructs. FACS analysis demonstrated the expression of αVβ3, α6β1 and α9β1 integrins in xenograft cells. Treatment with bicistronic constructs reduced αVβ3, α6β1 and α9β1 integrin expressions in xenograft injected nude mice. Migration and invasion were also inhibited by MMP-9, uPAR and cathepsin B shRNA treatments as assessed by spheroid migration, wound healing, and Matrigel invasion assays. As expected, bicistronic constructs further inhibited the adhesion, migration and invasive potential of the xenograft cells as compared to individual treatments.

**Conclusions/Significance:**

Downregulation of MMP-9, uPAR and cathespin B alone and in combination inhibits adhesion, migration and invasive potential of glioma xenografts by downregulating integrins and associated signaling molecules. Considering the existence of integrin inhibitor-resistant cancer cells, our study provides a novel and effective approach to inhibiting integrins by downregulating MMP-9, uPAR and cathepsin B in the treatment of glioma.

RETRACTED

## Introduction

Integrins are a family of adhesion molecules involved in interactions between the cell and the surrounding extracellular matrix (ECM). Although the classic role of integrins is to anchor cells to the ECM, they are known to participate in a variety of signaling pathways and to play important roles in fetal development, morphogenesis, cell migration, wound healing, and malignant transformation [1]–[6]. The heterodimerization of 19α-integrin and 8β-integrin subunits is thought to yield 25 integrin αβ heterodimers, which form receptors for an overlapping group of ECM molecules in almost every cell type [7]. Through interactions with the ECM, integrins control many cellular processes that occur in the progression of diseases such as cancer. Integrin signaling regulates diverse functions in tumor cells, including migration, invasion, proliferation and survival. In several tumor types, the expression of particular integrins correlates with increased disease progression and decreased patient survival [8].

Glioblastoma multiforme (GBM) is a highly malignant neoplasm of central nervous system. Strategies to treat infiltrating gliomas, such as chemotherapy and gene therapy, have remained largely unsuccessful and the property that makes glioma resistant to treatment is the tendency of the tumor cells to invade normal brain tissue [9]. Invasiveness is thus considered to be a major determinant of the malignant behavior of human gliomas. Integrins, the family of adhesive receptors promote the invasiveness of glioma. The role of integrins in cell migration and invasion is one of their most studied functions in tumor biology [10], [11]. Integrins directly bind components of the ECM and provide the traction necessary for cell motility and invasion. ECM remodeling is also controlled by integrins, which regulate the localization and activity of proteases. Proteases involved in these processes include serine proteases (the plasminogen activators uPA and tPA), matrix metalloproteinases (MMPs), and cysteine proteases (cathepsins B, D, L and H) [12].

GBM cells secrete MMPs and their mRNA and protein levels are elevated in patient biopsy tissues [13]–[15]. Significant correlation between MMP-9 levels and the histological grade of malignancy has been reported [16]. Furthermore, interactions between integrins expressed by glioma cells and the ECM and the activity of MMPs form the basis for glioma cell migration and invasion [17]. Expression of urokinase-type plasminogen activator receptor (uPAR) is much more robust in high-grade than in low-grade human gliomas [18]. Localization of uPAR mRNA in astrocytoma cells and the endothelial cells within brain tumor tissue has been reported and the expression of uPAR in the invading astrocytoma cells appears to have a critical role in the invasive behavior of glioblastoma [18]. Despite the controversy surrounding whether uPAR and integrins interact directly, many studies show that uPAR signaling requires integrin co-receptors. Furthermore, some non-integrin co-receptors of uPAR cooperate with integrins in signaling or influence uPAR-integrin interactions [19], [20]. Additionally, uPA-uPAR binding results in the expression of cathepsin B [21], another important protease involved in ECM degradation, and significantly higher levels of cathepsin B has been found in high-grade glioblastomas [22], [23].

RETRACTED

Taken together, the proteases MMP-9, uPA and Cathepsin B play critical roles in glioma pathology and have the combined ability to break down the ECM components. Moreover, the expression of one protease has a direct or indirect influence on the expression of other proteases. As such, the net proteolytic, and therefore invasive, potential of a given tumor cell might depend on the interplay between many proteolytic enzymes. In this scenario, targeting only one protease will definitely not result in the expected therapeutic outcome. Hence, in the present study, we investigated the effect of downregulating MMP-9, uPAR and ctahepsin B using both single as well as MMP-9/uPAR and MMP-9/cathepsin B bicistronic shRNA plasmid constructs on the expression of integrins and on the migrating and invasive potential of glioma xenograft cells.

## Results

### Effect of shRNA constructs on MMP-9, uPAR, and cathepsin B

Gelatin zymography revealed an inhibition of MMP-9 activity with all the treatments (Fig. 1A). The activity/expression of one protease has a direct or indirect influence on the activity/expression of other proteases. Our results were also in agreement with this fact and hence we noticed a prominent reduction in MMP-9 activity not only with M-sh treatment in 4910 cells but also with other treatments. In addition, fibrin zymography revealed prominent reductions in uPA activity with all the treatments in 4910 cells (Fig. 1A) and further supported the fact that activity/expression of one protease influence the activity/expression of other proteases and related molecules. Western blot analysis results clearly demonstrated significant reductions in protein expressions of these molecules with all the treatments except SV-sh compared to control cells (Fig. 1A–B). RT-PCR analysis of the cDNAs obtained from control and transfected 4910 cells revealed similar kind of reductions in these molecules at mRNA level (Fig. 1A). Taken together, these experiments at activity, protein and mRNA levels clearly demonstrate the efficiency of the shRNA plasmid constructs and the appropriate transfection conditions in xenograft cells. Reduction in the mRNA levels of MMP-9, uPAR and cathepsin B in M-sh, U-sh and C-sh transfected 4910 cells indicated a downregulation of MMP-9, uPAR and cathespin B target mRNAs, the mechanism by which shRNAs are proposed to work [24], [25]. Bands related to GAPDH at mRNA and protein levels associated with various treatments in 4910 cells indicate that similar amounts of mRNA/protein were loaded in all treatment groups.

RETRACTED

**Figure 1:** Efficiency of shRNA plasmid constructs and their effect on adhesion of xenografts to various ECM proteins. (A) Activity, protein and mRNA expressions of MMP-9, uPAR and cathepsin B in 4910 xenograft cells. MMP-9 and uPA activity was determined by gelatin and fibrin zymography after treatments with scrambled vector (SV-sh), MMP-9 (M-sh), uPAR (U-sh), cathepsin B (C-sh), MMP-9/uPAR (MU-sh) and MMP-9/cathepsin B (MC-sh) plasmid shRNAs. Western blot analysis showing MMP-9, uPAR and cathepsin B protein expression levels were reduced after M-sh, U-sh, C-sh, MU-sh and MC-sh treatments. n = 3. RT-PCR of 4910 cells transfected with SV-sh, M-sh, U-sh, C-sh, MU-sh and MC-sh was performed as per standard protocols. Further, quantification of the Western blots (B) revealed significant reductions in protein expressions after M-sh, U-sh, C-sh, MU-sh and MC-sh treatments. n = 3. Values shown are the mean (±SEM). *p<0.05 vs. control (C) Adhesion assay was performed to evaluate the effect of SV-sh, M-sh, U-sh, C-sh, MU-sh and MC-sh treatments in 4910 and 5310 glioma xenograft cells on their adhesive potential to collagen (type I), vitronectin, fibronectin and laminin coated plates. Percent adhesion was calculated from the mean obtained from 3 independent experiments and values shown are the mean (±SEM). *p<0.05 vs. control.

### Downregulation of proteases and uPAR inhibits adhesion to ECM proteins

Cell adhesion to ECM is a crucial regulator of many functions, including cell cycle, survival, migration, proliferation, differentiation and ultimately, tumor invasion [4], [26]. All the treatments (M-sh, U-sh, C-sh, MU-sh and MC-sh) inhibited the adhesion of both the xenografts to collagen, vitronectin, fibronectin and laminin. M-sh, U-sh and C-sh treatments in these xenografts significantly inhibited their adhesion to collagen (M-sh-39%, U-sh-51% and C-sh-57% inhibition in 4910 cells and M-sh-40%, U-sh-44% and C-sh-59% inhibition in 5310 cells), vitronectin (M-sh-51%, U-sh-45% and C-sh-57% inhibition in 4910 cells and M-sh-56%, U-sh-58% and C-sh-58% inhibition in 5310 cells), fibronectin (M-sh-36%, U-sh-48% and C-sh-48% inhibition in 4910 cells and M-sh-30%, U-sh-37% and C-sh-41% inhibition in 5310 cells), and laminin (M-sh-50%, U-sh-34% and C-sh-45% inhibition in 4910 cells and M-sh-48%, U-sh-52% and C-sh-65% inhibition in 5310 cells) (Fig. 1C). As expected, downregulation of MMP-9 in combination either with uPAR or cathepsin B further inhibited the adhesion of 4910 and 5310 cells to collagen, vitronectin, fibronectin and laminin (Fig. 1C). Results of the adhesion assay suggest bicistronic constructs that can simultaneously downregulate two molecules are more effective in reducing the adhesion of xenografts to various ECM proteins when compared to the single constructs that can only downregulate one molecule at a time. Interestingly, MC-sh treatment was found to be more effective than MU-sh in reducing the adhesion of both the xenografts to collagen and vitronectin.

RETRACTED

Integrins are transmembrane receptors for ECM proteins such as collagen, fibronectin, vitronectin and laminin. The classic role of integrins is to anchor cells to the ECM. Upregulation of α2β1, α3β1, α5β1, α6β1, αVβ3 and α9β1 integrins in glioblastoma was previously reported [27]–[29]. Hence, in the present study, we assessed the effect of downregulating uPAR, MMP-9 and cathepsin B alone and in combination on integrin expression. Although we have performed RT-PCR analysis by using several alpha and beta integrin primers, here we presented/discussed only those integrins that are affected in 4910 cells with shRNA treatments. All the affected integrins in 4910 cells were tested in 5310 cells and subjected to all the shRNA treatments. RT-PCR analysis of β1 and β3 integrins in 4910 and 5310 xenografts treated with various shRNAs for MMP-9, uPAR and cathepsin B revealed a marked reduction in their respective mRNA expression levels as compared to the controls (Fig. 2A). All the treatments downregulated the mRNA levels of β1 and β3 in both the xenografts except β1 and β3 mRNA levels in M-sh-treated 4910 xenograft cells. However, a significant reduction in these β integrin mRNA levels was noticed in both the xenografts treated with bicistronic constructs that simultaneously downregulate MMP-9 and either uPAR or cathespin B (Fig. 2A). The mRNA levels of several alpha integrins were reduced with MMP-9, uPAR and cathepsin B downregulation (Fig. 2B). α6, α9 and αV mRNA levels were downregulated in both the xenograft cell lines under all the treatment conditions.

RETRACTED

**Figure 2:** RT-PCR analysis of integrins. (A) RT-PCR analysis of 4910 and 5310 cells transfected with scrambled vector (SV-sh), MMP-9 (M-sh), uPAR (U-sh), cathepsin B (C-sh), MMP-9/uPAR (MU-sh) and MMP-9/cathepsin B (MC-sh) plasmid shRNAs, showing the mRNA expressions of β integrins (β1 and β3) (A) and α integrins (α1, α2, α6, α7, α9, α10, and αV) (B).

Immunocytochemistry of β1 and β3 integrins in 4910 and 5310 xenografts subjected to various shRNA treatments revealed a marked reduction in their protein expressions with all the treatments (Fig. 3A). Transfection with a scrambled vector in either of the xenografts did not affect the expression of these integrins. Reductions in the protein expressions similar to mRNA levels were noticed with α6, α9 and αV integrins when the transfected cells were subjected to immunocytochemistry (Fig. 3B). α1, α2, α7 and α10 integrins were downregulated only in 4910 xenograft cells treated with U-sh, C-sh, MU-sh and MC-sh (data not shown). These findings were further strengthened by the immunoblot analysis results wherein αV, α6, α9, β1 and β3 integrin protein expressions were significantly reduced after MU-sh and MC-sh treatments in 4910 cells (Fig. 4A–B). Based on these results and the earlier reported data [27]–[29], we hypothesize the involvement of αVβ3, α6β1 and α9β1 heterodimer combinations on the effects mediated by our shRNA treatments in the glioma xenografts studied in this present investigation. FACS analysis results clearly demonstrated that 4910 cells express α6β1, α9β1 and αVβ3 integrin heterodimers (Fig. 4C). Immunohistochemical analysis performed on the slide tissue microarrays of clinical GBM samples revealed the presence of αVβ3, α6β1 and α9β1 integrins on several GBM clinical samples compared to normal cerebrum (Fig. 4D).

**Figure 3:** Effect of shRNA plasmid constructs on the expression of integrins at protein level. (A) Immunocytochemistry was performed to evaluate the effect of various shRNA treatments on the expressions of β1 and β3 integrins. Microscopic images demonstrate β1 and β3 integrin expressions (red fluorescence) in 4910 and 5310 cells transfected with scrambled vector (SV-sh), MMP-9 (M-sh), uPAR (U-sh), cathepsin B (C-sh), MMP-9/uPAR (MU-sh) and MMP-9/cathepsin B (MC-sh). All treatments reduced β1 and β3 integrins expression. (B) The effect of various shRNA treatments on the expressions of α6, α9 and αV integrins was also evaluated and the microscopic images demonstrate α6, α9 and αV integrins expression in 4910 and 5310 cells transfected with SV-sh, M-sh, U-sh, C-sh, MU-sh and MC-sh. All the treatments reduced α6, α9 and αV integrins expression in both the cell lines.

**Figure 4:** Effect of bicistronic constructs on integrins and the expression of αVβ3, α6β1 and α9β1 integrins on glioma xenografts and GBM clinical samples. (A) Western blot analysis depicting the reduced protein expressions of αV, α6, α9, β1 and β3 integrins after MMP-9/uPAR (MU-sh) and MMP-9/cathepsin B (MC-sh) plasmid shRNA treatments in 4910 cells. n = 3. Further, quantification of the Western blots (B) revealed significant reductions in protein expressions after MU-sh and MC-sh treatments. n = 3. Values shown are the mean (±SEM). *p<0.05 vs. control. (C) FACS analysis showing the presence of αVβ3, α6β1 and α9β1 integrin heterodimers on 4910 glioma xenogaft cells. 4910 cells, in which iso match mouse IgG used as the primary antibody served as negative controls. NC-negative control (D) Immunohistochemistry of normal cerebrum and glioblastoma multiforme (GBM) for αVβ3, α6β1 and α9β1 integrin heterodimer expressions. GBM tissue micro arrays were processed for immunohistochemistry. Prominent brown staining indicative of αVβ3, α6β1 or α9β1 integrin expression was noticed in GBM samples. Scale bar = 100 µm.

RETRACTED

### shRNA treatment inhibited the migrating and invasive potential of glioma xenografts

In control and SV-sh-treated xenografts, 80–90% of the wound repair occurred within 16 h after creating the wound in 5310 and 4910 cells. Hence, the percent wound repair after treatments with M-sh, U-sh, C-sh, MU-sh and MC-sh was assessed at 16 h time point in 5310 and 4910 cells (Fig. 5A). We noticed significant reduction in percent wound repair with all the treatments in both the xenografts. Quantification of the results revealed that the wound reduced to 38%, 57%, 54%, 29% and 1% in 5310 and 51%, 54%, 45%, 43% and 32% in 4910 cells treated with M-sh, U-sh, C-sh, MU-sh and MC-sh, respectively (Fig. 5C). As assessed by spheroid migration assay, downregulating individual molecules using M-sh, U-sh and C-sh reduced migration of cells from the spheroids (Fig. 5B). Significant and prominent reductions in migration of the cells from spheroids were noticed upon treatment with bicistronic constructs MU-sh and MC-sh (Fig. 5D). Quantification of migration of the cells from spheroids revealed 67%, 83%, 58%, 61% and 23% reduction in 4910 and 50%, 53%, 50%, 38% and 30% reduction in 5310 cells treated with M-sh, U-sh, C-sh, MU-sh and MC-sh, respectively (Fig. 5D). The most dangerous feature of malignancy is invasive and metastatic potential. Simultaneous downregulation of MMP-9 along with either uPAR or cathepsin B reduced the invasive potential of 4910 and 5310 cells through the Matrigel (Fig. 5E). Quantification of Matrigel invasion assay results revealed a significant reduction in invasive potential of xenografts when subjected to treatment with either of the bicistronic constructs (Fig. 5F).

RETRACTED

**Figure 5:** Wound healing, spheroid migration and Matrigel invasion assays. (A) Reduction in wound healing indicative of reduced migration potential was noticed after treatments with MMP-9 (M-sh), uPAR (U-sh), cathepsin B (C-sh), MMP-9/uPAR (MU-sh) and MMP-9/cathepsin B (MC-sh) plasmid shRNAs in both 4910 and 5310 cells. Untreated and SV-sh transfected cells served as controls. (B) Migration of the cells from 4910 and 5310 spheroids transfected with M-sh, U-sh, C-sh, MU-sh and MC-sh was prominently reduced. (C, D) Quantification of wound healing and spheroid migration assays. Percent wound repair was calculated from the mean of the average width of the wound obtained from 3 independent experiments. Similarly, percent migration was calculated from the mean of the average migration obtained from 3 independent experiments. Error bars indicate SEM. *p<0.05 vs. control. (E) Matrigel invasion assay of 4910 and 5310 cells transfected with SV-sh, MU-sh and MC-sh. MU-sh and MC-sh treatments prominently reduced the invasive potential of both 4910 and 5310 cells through Matrigel. (F) Invasion was quantified by counting the average number of invaded cells in five different fields with each treatment. Percent invasion was calculated from the mean of the average number of invaded cells obtained from 3 independent experiments. Error bars indicate SEM. *p<0.05 vs. control.

### Involvement of α9β1 on the migration potential of xenograft cells

Compared to αVβ3 and α6β1 integrins, very little is known about the role α9β1 integrin in glioma. We studied the effect of α9β1 blockade on the migratory potential of 5310 cells that are transfected with uPAR, MMP-9 and cathepsin B expressing plasmid DNAs. RT-PCR analysis of uPAR, MMP-9 and cathepsin B in 4910 and 5310 cells transfected with uPAR expressing (U-fl), MMP-9 expressing (M-fl) and cathepsin B expressing (C-fl) plasmid DNAs clearly demonstrated the efficiency of the constructs and transfections (Fig. 6A–B). As expected, significant increase in percent wound repair noticed with U-fl, M-fl and C-fl treatments in 5310 cells which was significantly blocked with the same treatments in presence of α9β1 antibody (Fig. 6C–D). Furthermore, α9β1 integrin levels as revealed by FACS analysis were significantly reduced after MU-sh and MC-sh treatments in 4910 cells (Fig. 6E). These results clearly demonstrate the involvement of α9β1 in uPAR, MMP-9 and cathepsin B mediated migration in glioma xenograft cells.

**Figure 6:** Involvement of α9β1 integrin on the migration potential of xenograft cells and the effect of bicistronic constructs on the glioma xenograft cell proliferation. (A) RT-PCR of 5310 and 4910 cells transfected with uPAR (U-fl), MMP-9 (M-fl), and cathepsin B (C-fl) expressing plasmid DNAs was performed as per standard protocols. Prominent increase in respective mRNA expressions noticed after U-fl, M-fl, and C-fl treatments. Further, quantification of the RT-PCR data (B) revealed significant increases in uPAR mRNA and MMP-9 mRNA expression after treatments with M-fl and C-fl, respectively in both the xenograft cells. (C) Wound healing indicative of increased migration potential noticed after treatments with U-fl, M-fl, and C-fl in 5310 cells was reduced with the same treatments in presence of α9β1 antibody. Photographs are the representative images obtained from three independent experiments. (D) Quantification of wound healing assay. Percent wound repair was calculated from the mean of the average width of the wound obtained from 3 independent experiments. Error bars indicate SEM. *p<0.05 vs. control. ^#^ *p*<0.05. (E) FACS analysis showing reduced α9β1 integrin levels in 4910 cells after MMP-9/uPAR (MU-sh) and MMP-9/cathepsin B (MC-sh) treatments. (F) Clonogeneic assay depicting the reduced proliferation of 4910 and 5310 cells after MU-sh and MC-sh treatments. After 14 days of incubation, the colonies containing more than 50 cells were counted. Images shown are the representatives obtained from three independent experiments. (G) MTT assay showing significant reduction in the proliferation of 4910 cells from Day 4 to Day 6 after MU-sh and MC-sh treatments. n = 3. *p<0.05 vs. control.

RETRACTED

### Effect of bicistronic constructs on proliferation *in vitro* and tumors *in vivo*

MU-sh and MC-sh treatments efficiently reduced the colony forming ability of 4910 and 5310 cells (Fig. 6F). Similarly, proliferation of 4910 cells as evidenced by MTT assay was significantly reduced on Days 4, 5 and 6 after MU-sh and MC-sh treatments compared to untreated 4910 cells (Fig. 6G).

Hematoxylin and eosin staining performed on mouse brains (injected with xenograft cells 2 weeks before treatment) revealed a prominent reduction of tumor growth in MU-sh and MC-sh treated mouse brains when compared to the controls (Fig. 7A). Aggressive tumor formation was noticed in xenografts injected mouse brains compared to normal brains (Fig. 7A–B). Furthermore, the apoptotic index of tumor cells quantified by the number of positive cells for TUNEL staining showed a drastic and significant increase in the number of apoptotic cells in the tumor sections from mice that were treated with bicistronic constructs (data not shown). Brains of the animals that were sacrificed 2–3 weeks prior to the end of the treatment were used to evaluate the effect of MU-sh and MC-sh treatments on the expression of αVβ3, α6β1 and α9β1 integrins. As expected, prominent reduction of αVβ3, α6β1 and α9β1 integrin expression was noticed on the 5310 *in vivo* tumors that were treated with MU-sh and MC-sh (Fig. 7C). Immunohistochemical analysis of platelet endothelial cell adhesion molecule (PECAM-1) performed on the brain sections of 4910 and 5310 control tumors and MU-sh and MC-sh treated 5310 tumors (from the animals that are sacrificed 2–3 weeks prior to the end of the treatment) revealed that the extent of blood vessels in 4910 and 5310 untreated tumors are more compared to MU-sh and MC-sh treated 5310 tumors (Fig. 7D).

RETRACTED

**Figure 7:** Effect of treatment with bicistronic constructs on the brain tumors in nude mice pre-injected with xenograft cells. (A) shRNA mediated regression of pre-established tumor growth. Hematoxylin and eosin staining performed on the brain sections obtained from various groups of animals revealed a prominent tumor reduction after MMP-9/uPAR (MU-sh) or MMP-9/cathepsin B (MC-sh) treatments. Each group consisted of 6 animals. Yellow curved line in 4910 and 5310 control brain sections indicate the tumor area. (B) Normal nude mice brain section stained with hematoxylin and eosin. (C) Immunohistochemical comparison of control, MU-sh and MC-sh-treated nude mice which are pre-injected with 5310 cells (and sacrificed 2–3 weeks prior to the end of the treatment), to analyze the expression of αVβ3, α6β1 and α9β1 integrin heterodimers. Brown staining indicative of αVβ3, α6β1 or α9β1 integrin expression was reduced in MU-sh and MC-sh treated sections compared to controls. n = 6. Scale bar = 50 µm. (D) Untreated 4910 and 5310 *in vivo* tumors were prominently stained for platelet endothelial cell adhesion molecule (PECAM-1) whereas the intensity of brown staining was reduced in 5310 *in vivo* tumors after MU-sh and MC-sh treatments.

### Effect of silencing proteases and uPAR on FAK and other migration molecules

Our results clearly demonstrated the involvement of αVβ3, α6β1 and α9β1 and integrins in the effects mediated by shRNA treatments and thereby affected the adhesive, migrating and invasive potential of glioma xenografts. To further confirm the integrins involvement, we sought to determine the effect of these shRNA treatments on the signaling molecules associated with integrin mediated migration. Hence, we evaluated the effect of MU-sh and MC-sh treatments on several molecules such as FAK, talin1, talin2, profilin, vinculin, actinin, tensin, Rac1 and Arp2 in both the xenograft cell lines by using RT-PCR analysis. Downregulation of FAK, talin1, talin 2, profilin, tensin and Arp2 was noticed in treated 5310 cells whereas in 4910 cells, FAK, talin1, talin2, vinculin, actinin, tensin and Arp2 levels were reduced with both MU-sh and MC-sh treatments (Fig. 8A). Rac1 mRNA levels reduced only in MC-sh treated 5310 cells. Further, vinculin and actinin mRNA levels reduced only in 4910 cells treated with these bicistronic constructs. The expressions of FAK, phospho-FAK, cSrc, phospho-Src, Arp2, F-actin, paxillin, phospho-paxillin at protein level were reduced with both MU-sh and MC-sh treatments in 5310 cells (Fig. 8B). Rac1, talin1, α-actinin and vinculin protein expressions were reduced only in MC-sh treated 5310 xenografts. MU-sh and MC-sh treatments did not affect cofilin levels. In agreement with our adhesion, migration and invasion assay results, a more pronounced downregulation was noticed in majority of the migration-related molecules with MC-sh as compared to MU-sh.

RETRACTED

**Figure 8:** RT PCR and Western blot analysis of the molecules associated with integrin-mediated migration. (A) RT-PCR of 4910 and 5310 glioma xenograft cells transfected with scrambled vector (SV-sh), MMP-9/uPAR (MU-sh) and MMP-9/cathepsin B (MC-sh) plasmid shRNAs was performed as per standard protocol described in materials and methods. Several genes were downregulated with MU-sh and MC-sh treatments in both the xenograft cells. Results presented are the representative images of three independent experiments. (B) Western blot analysis showing the effect of bicistronic constructs (MU-sh and MC-sh) on the protein expressions of FAK, p-FAK (Tyr397), cSrc, p-Src (Tyr527), Rac1, Arp2, F-actin, talin1, paxillin, p-paxillin (Tyr118), α-actinin, cofilin and vinculin in 5310 human glioma xenograft cells. The expressions of majority of the proteins associated with integrin-mediated migration were reduced with MU-sh and MC-sh treatments. n = 3.

## Discussion

Malignant gliomas are highly invasive neoplasms. They may make a permissive environment for invasion by synthesizing and depositing an autologus matrix that facilitates their own motility. The ECM, which is a key component of the tissue destroyed during tumor cell invasion, is a dynamic environment that has a pivotal role in regulating cellular functions during pathological remodeling processes, such as tumor invasion and metastasis. Tumor ECM and basement membranes of tumor blood vessels have shown tenacin, vitronectin, collagens, fibronectin, laminin, hyaluronan, chondroitin sulfate and heparan sulfate. Collagen, laminin, tenacin, fibronectin and vitronectin serve as permissive substrates for glioma cell migration. Cell adhesion plays a major role in regulating cell movement. Adhesion of glioma xenograft cells to various components of ECM such as collagen, vitronectin, fibronectin and laminin was significantly inhibited by MMP-9, uPAR and cathepsin B shRNA plasmid constructs. Simultaneous targeting of multiple molecules has been more synergistic than additive [30]. As expected, inhibition of adhesion of these cells to ECM components is much more significant with the simultaneous downregulation of MMP-9 and uPAR or MMP-9 and cathepsin B.

RETRACTED

Integrins expressed in tumor cells contribute to tumor progression and metastasis by increasing tumor cell migration, invasion, proliferation and survival [8]. Integrin adhesion to ECM provides the traction required for tumor cell invasion. Interactions and signaling mechanisms among uPAR, MMP-9 and cathepsin B associated with integrin involvement were well studied and reported [31]–[34]. Integrins are essential uPAR signaling co-receptors and the interactions between uPAR/β1 and uPAR/β3 have an important role in signaling for cell migration and invasion [34]. It was reported that the cleavage of αV integrin subunit precursor by MMP-14 enhanced cancer-cell migration [35]. Further, cooperation between MMP-9 and integrins is known to activate αVβ3, which strongly enhanced tumor migration [36]. Cathepsin B is known to be associated with uPAR and its integrin-mediated signaling ability [37]. Moreover, immunoprecipitation of the 4910 and 5310 glioma xenograft cell lysates with β1 integrin followed by immunoblot analysis with cathepsin B indicated a possibility for the direct or indirect interaction between these two molecules (data not shown). Inhibition of adhesion by MMP-9, uPAR and cathepsin B silencing in the present study resulted in a significant reduction in the expressions of several alpha and beta integrins both at mRNA and protein levels. αV, α6, α9, β1 and β3 integrin mRNA and protein expressions were prominently downregulated in both the xenograft cell lines with all the treatments. Upregulation of α2β1, α3β1, α5β1, αVβ3 and α6β1 integrins on GBM have already been reported [28], [29]. In 2008, deHart et al., identified that α9β1 integrin increase cell migration by modulation of polyamine metabolism and activation of potassium channels [38]. Unlike other integrin heterodimers, α9β1 was able to both increase cell migration and inhibit cell spreading [39], [40]. It was recently found that α9β1 integrin played a significant role in the progression of glioblastoma [27]. Hence, we expected the involvement of αVβ3, α6β1 and α9β1 heterodimer combinations on the effects mediated by our shRNA treatments in the xenografts studied in our present investigation. FACS analysis confirmed the expression of αVβ3, α6β1 and α9β1 integrins on xenograft cells. Bicistronic constructs significantly reduced α9β1 levels *in vitro* in 4910 cells. These constructs also reduced the proliferation of xenograft cells *in vitro*. *In vivo* studies in nude mice injected with 5310 cells revealed a prominent reductions in the expression of integrin heterodimers (αVβ3, α6β1 and α9β1) when treated with MMP-9/uPAR or MMP-9/cathepsin B shRNAs. Furthermore, drastic reductions in tumor growth and extent of blood vessels in tumor mass (neoangiogenesis) were noticed *in vivo* after MU-sh and MC-sh treatments in xenograft cells injected nude mice. These results are in agreement with our earlier reports, wherein we have noticed a significant decrease in tumor growth with MU-sh and MC-sh treatments in SNB19 cells injected mouse brains [33], [41].

α9β1 has distinguished its functionality from other integrins (αVβ3 and α3β1) by facilitating accelerated cell migration [42]. Hence, in the present study, we performed spheroid migration assay and wound healing assay in order to address the effect of silencing proteases on migratory potential of glioma xenografts. All the treatments with single (M-sh, U-sh and C-sh) and bicistronic constructs (MU-sh and MC-sh) significantly reduced the migration of glioma xenografts in all the above-mentioned assays. Our results clearly revealed that the bicistronic constructs were more effective than the single constructs in reducing the migrating potential of glioma xenografts. Further, in concurrence with adhesion assay results, we have noticed a marked reduction in migration in all the assays with MC-sh as compared to MU-sh. Integrin α9β1 is classified within a two member sub-family of integrins highlighted in part by its specialized role in cell migration [43]. Unlike other integrins, α9β1 has been proposed to utilize inducible nitric oxide synthase (iNOS)-nitric oxide (NO) and spermidine/spermine acetyl transferase (SSAT)-inward rectifier potassium channel (Kir) pathways along with common integrin signaling proteins such as Src and FAK to transduce cell migration [43]. Significant inhibition of uPAR, MMP-9 and cathepsin B mediated migration in 5310 xenograft cells by α9β1 integrin blockade, clearly demonstrated its possible role. Gliomas are highly invasive and the invasive nature of gliomas has an important role in the ineffectiveness of current treatment modalities, as the remaining cancer cells inevitably infiltrate the surrounding normal brain tissue and lead to tumor recurrence [37]. Hence, we felt it is crucial to evaluate the effect of shRNA treatments on the invasive potential of xenografts and as expected, the MU-sh and MC-sh treatments significantly inhibited the invasion of both 4910 and 5310 cells through the Matrigel.

RETRACTED

In this study, downregulation of uPAR and the proteases, MMP-9 and cathepsin B showed a significant reduction in the adhesion, migration and invasive potential of xenografts and also affected the levels of several alpha and beta integrins. Like other integrins α9β1 ligation can activate signaling through Src and FAK mediated tyrosine phosphorylation of multiple proteins including p130Cas and paxillin [40], [44]. Hence, we suspected that our treatments played a significant role in regulating the molecules associated with integrin-mediated signaling that leads to migration. Focal adhesion kinase (FAK) is a cytoplasmic tyrosine kinase that has been implicated to play a key role in integrin-mediated signal transduction pathways [5], [45]. The most important transmembrane receptors associated with uPAR signaling are the integrin family of ECM receptors [34]. uPAR/β1 integrin interactions are frequently associated with the activation of FAK and ERK, whereas uPAR/β3 integrin interactions are associated with the activation of Rac [20], [46]–[48]. Prominent reduction in FAK mRNA levels with MU-sh and MC-sh treatments in both the xenograft cell lines in the present study demonstrated the involvement of integrins via FAK in inhibiting their adhesion and migration potential. Even though the migration potential of both the xenografts was significantly reduced with all the shRNA treatments, they behaved differently in regulating the mRNA expressions of various genes associated with migration. Reduced FAK, phospho-FAK, cSrc, phospho-Src, Arp2, F-actin, paxillin, phospho-paxillin protein levels after treatment with bicistronic constructs in 5310 cells further strengthened our hypothesis that our treatments inhibit the migratory potential of these xenografts.

Taken together, our findings clearly demonstrated that shRNA-mediated silencing of MMP-9, uPAR, and cathepsin B inhibited adhesive, migrating and invasive potentials of glioma xenografts. Bicistronic constructs that can simultaneously downregulate MMP-9 and uPAR or MMP-9 and cathepsin B were more effective than any of the single constructs. We also show the involvement of several integrins, FAK and associated molecules in the effects mediated by our shRNA constructs. Furthermore, for the first time, we have shown the involvement of α9β1 integrin in the effects mediated by MMP-9, uPAR and cathepsin B silencing in glioma xenografts. Considering the existence of integrin inhibitor-resistant cancer cells, our study provides a novel and effective approach for inhibiting integrins while downregulating MMP-9, uPAR and cathepsin B in treating glioma.

RETRACTED

## Materials and Methods

### Ethics Statement

The Institutional Animal Care and Use Committee of the University Of Illinois College Of Medicine at Peoria, Peoria, IL, USA approved all surgical interventions and post-operative animal care. The consent was written and approved. The approved protocol number is 851, dated November 20, 2009.

### Cell culture and transfection conditions

The xenograft cell lines (4910 and 5310) were kindly provided by Dr David James at University of California, San Francisco. These xenografts were generated and maintained in mice and are highly invasive in mouse brain [49]. 4910 and 5310 xenografts were maintained in RPMI 1640, supplemented with 10% fetal bovine serum, 50 μg/ml streptomycin and 50 U/ml penicillin in a humidified atmosphere containing 5% CO_2_ at 37°C. Xenografts were transfected with SV-sh (scrambled vector), M-sh (MMP-9), U-sh (uPAR), C-sh (cathepsin B), MU-sh (MMP-9 and uPAR) or MC-sh (MMP-9 and cathepsin B) shRNA expressing plasmids using Fugene® HD reagent (Roche Diagnostics, Indianapolis, IN) as per the manufacturer's instructions. After transfection, cells were incubated in serum-containing medium for a minimum of 60 h.

### Construction of shRNA and gene expressing plasmids

Plasmid shRNAs for MMP9, uPAR, cathespin B, MMP-9/uPAR and MMP-9/CathespinB designed in our laboratory [31], [41], [50] were used to transfect the xenograft cells. Briefly, a pCDNA-3 plasmid with a human cytomegalovirus (CMV) promoter was used to construct the shRNA-expressing vectors. A pCDNA3-scrambled vector with an imperfect sequence, which does not form a perfect hairpin structure, was used as a control (SV-sh). MMP-9 expressing (M-fl) plasmids in pDNR-CMV vector were designed and constructed in our laboratory whereas uPAR expressing (U-fl) and cathepsin B expressing (C-fl) plasmids were purchased from Origene (Rockville, MD).

### Antibodies

Several antibodies were used in various techniques such as Western blot, immunocytochemistry, immunohistochemistry and fluorescent-activated cell sorting (FACS) analysis while determining the changes in protein expression associated with various treatments. Antibodies targeting MMP-9, β3 integrin, α6 integrin, α9 integrin, α9β1 integrin, PECAM-1, FAK, Phospho FAK (Tyr 397), cSrc, talin1, vinculin were obtained from Santa Cruz Biotechnology (Santa Cruz, CA); Phospho Src (Tyr 527), Arp2, paxillin, phospho paxillin, cofilin were obtained from Cell Signaling (Boston, MA); β1 integrin, α6β1 integrin, αVβ3 integrin were obtained from Millipore (Billerica, MA); uPAR was obtained from R&D Systems (Minneapolis, MN); α-actinin was obtained from Sigma (St. Louis, MO); cathepsin B was obtained from Athens Research and Technology (Athens, GA); αV integrin, F-actin were obtained from Abcam (Cambridge, MA); αVβ3 integrin, Rac1 were obtained from BD Biosciences (San Jose, CA); and glyceraldehyde-3-phosphate dehydrogenase (GAPDH) was obtained from Novus Biologicals (Littleton, CO).

RETRACTED

### Gelatin zymography

MMP-9 activity in the conditioned medium was determined by gelatin zymography. 4910 and 5310 human glioma xenograft cells were transfected with SV-sh, M-sh, U-sh, C-sh, MU-sh and MC-sh for 72 h. Cells were washed and incubated with serum-free medium overnight. Equal amounts of protein were electrophoresed in 10% SDS-polyacrylamide gels containing 1.5 mg/mL gelatin. The gels were washed and gently shaken in three consecutive washings in 2.5% Triton X-100 solution to remove SDS. The gels were then incubated at 37°C overnight in incubation buffer [50 mmol/l Tris-HCl (pH 7.5), 0.05% NaN3, 5 mmol/l CaCl2 and 1 μmol/l ZnCl2]. Next, the gels were stained with 0.1% amido black in 10% acetic acid and 10% isopropanol and subsequently destained for 1 h. Gelatinolytic activities were identified as clear zones of lysis against a dark background.

### Fibrinogen zymography

4910 and 5310 human glioma xenograft cells were transfected with SV-sh, M-sh, U-sh, C-sh, MU-sh or MC-sh for 72 h. Cells were washed and incubated with serum-free medium overnight. Conditioned media was collected and zymography was performed to determine uPA activity. Equal amounts of protein samples were resolved on 10% SDS-polyacrylamide gels containing plasminogen and fibrinogen and stained with 0.1% amido black in 10% acetic acid and 10% isopropanol and subsequently destained for 1 h.

### Western blot analysis

Xenograft cells were transfected with SV-sh, M-sh, U-sh, C-sh, MU-sh or MC-sh for 72 h. Cells were collected and lysed in RIPA buffer [50 mmol/ml Tris-HCl (pH 8.0), 150 mmol/ml NaCl, 1% IGEPAL, 0.5% sodium deoxycholate, 0.1% SDS] containing 1 mM sodium orthovanadate, 0.5 mM PMSF, 10 µ/ml aprotinin, 10 μg/ml leupeptin and resolved via SDS-PAGE. After overnight transfer onto nitrocellulose membranes, blots were blocked with 5% non-fat dry milk in PBS and 0.1% Tween-20. Blots were then incubated with primary antibody, followed by incubation with HRP-conjugated secondary antibody. Immunoreactive bands were visualized using chemiluminescence ECL Western blotting detection reagents on Hyperfilm-MP autoradiography film (Amersham, Piscataway, NJ). GAPDH (housekeeping gene) antibody was used to verify that similar amounts of protein were loaded in all lanes.

### Reverse transcription PCR analysis

4910 and 5310 cells were transfected with SV-sh, M-sh, U- sh, C-sh, MU-sh, MC-sh, U-fl, M-fl or C-fl. The cells were collected and total cell RNA was isolated. Approximately 500 ng of total RNA from each sample was synthesized into cDNA as per the manufacturer's instructions using the Transcriptor First Strand cDNA Synthesis Kit (Roche Diagnostics, Indianapolis, IN). We used the following sequences for the forward and reverse primers:

- for MMP-9, 5′CTCGAACTTTGACAGCGACA3′ (forward) and 5′GCCATTCACGTCGTCCTTAT3′ (reverse);
- for uPAR, 5′GCCTTACCGAGGTTGTGTGT3′ (forward) and 5′CATCCAGGCACTGTTCTTCA3′ (reverse);
- for cathepsin B, 5′GCTACAGCCCGACCTACAAA3′ (forward) and 5′CCAGTAGGGTGTGCCATTCT3′ (reverse);
- for integrin αV, 5′CACCAGCAGTCAGAGATGGA3′ (forward) and 5′GAACAACTGGCCCAACATCT3′ (reverse);
- for integrin α1, 5′GTCCAGTTGGGAGAGGTGAA3′ (forward) and 5′ACTTGAAATGTGGGGCTGAC3′ (reverse);
- for integrin α2, 5′CAAGTGGGATTCAGTGCAGA3′ (forward) and 5′GAGCACCAGCAACAAAGTGA3′ (reverse);
- for integrin α6, 5′CCCCGCTGGTTATAATCCTT3′ (forward) and 5′GGTTTCCTCCATGCACACTT3′ (reverse);
- for integrin α7, 5′GGGAACCAATACCCTGACCT3′ (forward) and 5′CTATAGCTGCTGGGGACTGC3′ (reverse);
- for integrin α9, 5′CGGAATCATGTCTCCAACCT3′ (forward) and 5′CTCTGCACCACCAGATGAGA3′ (reverse);
- for integrin α10, 5′CAACAGCATCTACCCCTGGT3′ (forward) and 5′GGTTCTTTGCTGCTCTCACC3′ (reverse);
- for integrin β1, 5′CATCTGCGAGTGTGGTGTCT3′ (forward) and 5′GGGGTAATTTGTCCCGACTT3′ (reverse);
- for integrin β3, 5′GCAATGGGACCTTTGAGTGT3′ (forward) and 5′GTGGCAGACACATTGACCAC3′ (reverse);
- for FAK, 5′AGCTGATTGGAGTCATCACAGA3′ (forward) and 5′GAGGGTAGGAGGACAATTTGG3′ (reverse);
- for talin1, 5′TGGAGAACTCAAAGGTGCTG3′ (forward) and 5′CGCCTTGATGGTCTTGACA3′ (reverse);
- for talin2, 5′CACACTGGATTTTGGGGAGT3′ (forward) and 5′ATATCCTGGCCGAGAGGTG3′ (reverse);
- for profilin, 5′AACGTTCGTCAACATCACG3′ (forward) and 5′TTTGGCAGCAATAAGGGGTA3′ (reverse);
- for vinculin, 5′TACGAAGACAGGGGAAAGGA3′ (forward) and 5′TTGGAGCTGAGATGCAAGTG3′ (reverse);
- for actinin, 5′GGCCAGTGATCTGTTGGAGT3′ (forward) and 5′TAGTCCTTCTGTCGCAGCAT3′ (reverse);
- for tensin, 5′AGACACCCCTGTCTGCTCTG3′ (forward) and 5′GGGAAACTCCCCACTGAAG3′ (reverse);
- for Rac1, 5′GGGAGACGGAGCTGTAGGTA3′ (forward) and 5′CAGCACCAATCTCCTTAGCC3′ (reverse);
- for Arp2, 5′CTTCTGTTGCGAGGATACGC3′ (forward) and 5′AAGTTTTTCCACATCACCCTTC3′ (reverse);
- for GAPDH, 5′AGCCACATCGCTCAGACACC3′ (forward) and 5′GTACTCAGCGGCCAGCATCG3′ (reverse);
- for β-actin, 5′GGCATCCTCACCCTGAAGTA3′ (forward) and 5′GGGGTGTTGAAGGTCTCAAA3′ (reverse);

Reverse transcriptase PCR was set up using the PCR cycle [95°C for 5 min, (95°C for 30 sec, 55–60°C for 30 sec, and 72°C for 30 sec)×30 cycles, 72°C for 10 min]. PCR products were resolved on a 1.6% agarose gel, visualized, and photographed under UV light.

RETRACTED

### Adhesion Assay

Adhesion was assessed as described previously [51] with modifications. 4910 and 5310 human glioma xenograft cells (1×10^6^) were seeded on 100-mm culture plates and incubated in a humidified atmosphere containing 5% CO_2_ at 37°C. 24 h after incubation, cells were transfected with SV-sh, M-sh, U-sh, C-sh, MU-sh or MC-sh. 72 h after transfection, cells were harvested by 50 mM EDTA treatment, washed with PBS, then resuspended in 10% serum-containing medium for 1 h at 37°C. Cells were washed twice with serum-free medium, resuspended in serum-free medium, and seeded at 30,000–50,000 cells/well in a 96-well plate coated with various components of extracellular matrix (ECM) such as collagen (type I), fibronectin, vitronectin or laminin. After 1–2 h incubation at 37°C, unattached cells were removed by rinsing the slides three times with PBS. The remaining attached cells were fixed and stained with Hema-3 (Fisher Scientific). Images in 5 different fields covering a majority of the area in each well of a 96-well plate were taken from all the treatment groups under a light microscope. The number of adhered cells from all the treatment groups was counted and the average was recorded for comparative quantification.

### Spheroid migration assay

4910 and 5310 spheroids were cultured in 96-well plates coated with 1% agar. Briefly, 3×10^4^ cells/well were seeded and cultured on a shaker at 100 rpm for 48 h in a humidified atmosphere containing 5% CO_2_ at 37°C. After the formation of spheroids, they were transfected with SV-sh, M-sh, U-sh, C-sh, MU-sh or MC-sh. 48 h after transfection, the spheroids were transferred to 24-well plates and incubated at 37°C. Twenty four hours after incubation, the spheroids were fixed and stained with Hema-3. Cell migration from the spheroids was assessed using light microscopy. The migration of cells from spheroids to monolayers was used as an index of cell migration and was measured using a microscope calibrated with a stage and ocular micrometer.

### Wound healing assay

To study cell migration, we seeded xenograft cells (4910 and 5310) at a density of 2×10^6^ in a 6-well plate and transfected the cells with SV-sh, M-sh, U-sh, C-sh, MU-sh or MC-sh for 72 h. Then, a straight scratch was made in individual wells with a 200 µL pipette tip. This point was considered the “0 h,” and the width of the wound was photographed under the microscope. After 6–16 h, the cells were checked for wound healing and photographed at 16 h under the microscope. Wound healing was measured by calculating the reduction in the width of the wound after incubation. We also studied the effect of U-fl, M-fl and C-fl treatments in the absence and presence of α9β1 antibody on migration in 4910 cells by performing this assay.

RETRACTED

### Matrigel invasion assay

4910 and 5310 cells were transfected with SV-sh, MU-sh or MC-sh for 72 h. Cells were trypsinized and 5×10^4^ cells were placed onto Matrigel-coated transwell inserts with 8-μm pore size. Cells were allowed to migrate through the Matrigel for 24 to 48 h. Then, cells in the upper chamber were removed with a cotton swab. The cells that adhered on the outer surface of the transwell insert and had invaded through the matrigel were fixed, stained with Hema-3, and counted under a light microscope as described previously [52].

### Immunocytochemistry

4910 and 5310 cells (1×10^4^) were seeded on 2-well chamber slides, incubated for 24 h, and transfected with SV-sh, M-sh, U-sh, C-sh, MU-sh or MC-sh for 72 h. Then, cells were fixed with 10% buffered formalin phosphate and incubated with 1% bovine serum albumin in PBS at room temperature for 1 h for blocking. After the slides were washed with PBS, primary antibodies were added at a concentration of 1∶100. The slides were incubated overnight at 4°C and washed thrice with PBS to remove excess primary antibody. Cells were then incubated with Alexa Fluor® 594 (goat anti-mouse IgG, red) fluorescent-labeled secondary antibody for 1 h at room temperature. The slides were then washed thrice with PBS and covered with glass coverslips, and fluorescent photomicrographs were obtained.

### Immunohistochemistry

Paraffin embedded brain sections (5 µm thick) from control and treatment groups were deparaffinized as per standard protocol. The sections were rinsed with PBS and treated with 1% BSA in PBS to prevent nonspecific staining and incubated with primary antibodies (1∶50 dilution) at 4°C overnight. The sections were then washed in PBS and incubated with appropriate HRP-conjugated secondary antibodies for 1 h at room temperature. After 1 h, sections were washed in PBS and incubated in DAB for 30 min. The slides were further washed with sterile water and subjected to dehydration. After dehydration, the slides were stained with hematoxylin to visualize the nucleus, mounted and observed under a light microscope. Immunohistochemical analysis for αVβ3, α6β1 and α9β1 integrins was performed on the slide tissue microarrays (obtained from US Biomax, Inc., Rockville, MD, USA) of clinical GBM samples.

### FACS analysis

4910 cells (2×10^6^) were seeded on 100-mm tissue culture plates, incubated for 48 h, and then treated with 50 mM EDTA, washed with PBS, pelleted at 1000 rpm for 5 min, and resuspended at a concentration of 1×10^6^ cells/mL in PBS. Cells were then incubated with HRP-conjugated or fluorescence conjugated primary antibodies for 1 h on ice, pelleted, and washed three times with PBS to remove excess primary antibody. Cells that were incubated with HRP-conjugated primary antibodies were then resuspended in 1 ml of PBS and incubated with Alexa Fluor® 594 (goat anti-mouse IgG, red) fluorescent labeled secondary antibody for 1 h on ice. After three more washes in PBS, cell pellet was resuspended in 10% buffered formalin and analyzed on a Coulter EPICS XL AB6064 flow cytometer (Beckman Coulter, Fullerton, CA). We also studied the effect of MU-sh and MC-sh treatments in 4910 cells on α9β1 integrin levels by performing FACS analysis.

RETRACTED

### Clonogenic assay

To study the effect of bicistronic plasmid shRNA treatments on proliferation, 4910 and 5310 cells were transfected with SV-sh, MU-sh or MC-sh. 72 h after transfection, cells were plated on 100-mm plates at 2000 cells per plate. Medium was subsequently changed every 3 days. After 2 weeks, the resulting colonies were fixed and stained with Hema-3, and counted as a measure of clonogenecity.

### Cell proliferation assay

Cell growth was assessed by MTT (3-(4,5-Dimethylthiazol-2-yl)-2,5-diphenyltetrazolium bromide) assay. 4910 cells were transfected with SV-sh, MU-sh or MC-sh. 72 h after transfection, 5×10^3^ cells were seeded in triplicate into 96-well plates and incubated different time intervals. Before each time point, we added 10 µl of 5 mg/ml freshly prepared MTT reagent to each well and continued the incubation for an additional 2 h to permit color development. After incubation, the crystals were dissolved in 2-propanol + hydrochloric acid solution and the plate was left in dark for 3 h. After 3 h, absorbance was measured using Biorad Microplate Reader.

### Intracranial administrations in nude mice

The Institutional Animal Care and Use Committee of the University Of Illinois College Of Medicine at Peoria, Peoria, IL, USA approved all surgical interventions and post-operative animal care. 4910 and 5310 xenografts were trypsinized and resuspended in serum free medium at a concentration of 0.2×10^5^ cells/µL. Nude mice were injected intracerebrally with a 10 µl aliquot (0.2×10^5^ cells/µL) under isofluorane anesthesia with the aid of a stereotactic frame. After two weeks, mice were separated into three groups in each cell line. The first, second and third groups served as the control, MU-sh-treated (150 µg), and MC-sh-treated (150 µg) groups respectively. MU-sh and MC-sh plasmid DNAs were injected into the brains of nude mice using Alzet mini pumps at the rate of 0.2 µL/h. The concentration of the plasmid solution was 2 µg/µL (100 µl per mouse, six mice in each group). After five weeks, the mice were sacrificed by intracardiac perfusion, first with PBS and then with 4% paraformaldehyde in normal saline. The brains were removed, stored in 4% paraformaldehyde, processed, embedded in paraffin, and sectioned (5 µm thick) using a microtome. Paraffin embedded sections were stained with hematoxylin and eosin to visualize tumor cells and to examine tumor volume.

RETRACTED

### Densitometry

Densitometry was performed using Image J Software (National Institutes of Health) to quantify the band intensities obtained from Western blot analysis and RT-PCR. Data represent average values from 3 separate experiments.

### Statistical analysis

Statistical comparisons were performed using Graph Pad Prism software (version 3.02). Quantitative data from Western blot analysis, RT-PCR, adhesion, migration and invasion assays was evaluated for statistical significance using one-way ANOVA. Bonferroni's post hoc test (multiple comparison tests) was used to compare any statistical significance between groups. Differences in the values were considered significant at *p*<0.05.
